# Cellular response to micropatterned growth promoting and inhibitory substrates

**DOI:** 10.1186/1472-6750-13-86

**Published:** 2013-10-11

**Authors:** Wiam Belkaid, Peter Thostrup, Patricia T Yam, Camille A Juzwik, Edward S Ruthazer, Ajit S Dhaunchak, David R Colman

**Affiliations:** 1 McGill Program in Neuroengineering, McGill University, Montreal, Canada; 2 Interdisciplinary Nanoscience Center, University of Aarhus, Aarhus, Denmark; 3 Montreal Neurological Institute, 3801 University St, Montreal, Quebec H3A 2B4, Canada; 4 Molecular Biology of Neural Development, Institut de Recherches Cliniques de Montréal, Montreal, Canada

**Keywords:** Microcontact printing, Polylysine, Myelin, Adhesion, Oli-neu, COS7, Primary culture

## Abstract

**Background:**

Normal development and the response to injury both require cell growth, migration and morphological remodeling, guided by a complex local landscape of permissive and inhibitory cues. A standard approach for studying by such cues is to culture cells on uniform substrates containing known concentrations of these molecules, however this method fails to represent the molecular complexity of the natural growth environment.

**Results:**

To mimic the local complexity of environmental conditions in vitro, we used a contact micropatterning technique to examine cell growth and differentiation on patterned substrates printed with the commonly studied growth permissive and inhibitory substrates, poly-L-lysine (PLL) and myelin, respectively. We show that micropatterning of PLL can be used to direct adherence and axonal outgrowth of hippocampal and cortical neurons as well as other cells with diverse morphologies like Oli-neu oligodendrocyte progenitor cell lines and fibroblast-like COS7 cells in culture. Surprisingly, COS7 cells exhibited a preference for low concentration (1 pg/mL) PLL zones over adjacent zones printed with high concentrations (1 mg/mL). We demonstrate that micropatterning is also useful for studying factors that inhibit growth as it can direct cells to grow along straight lines that are easy to quantify. Furthermore, we provide the first demonstration of microcontact printing of myelin-associated proteins and show that they impair process outgrowth from Oli-neu oligodendrocyte precursor cells.

**Conclusion:**

We conclude that microcontact printing is an efficient and reproducible method for patterning proteins and brain-derived myelin on glass surfaces in order to study the effects of the microenvironment on cell growth and morphogenesis.

## Background

The local microenvironment influences the growth and morphogenesis of developing cells in vivo [1,2]. Similarly, cultured cells respond to their local environment by regulating their adhesion, proliferation and differentiation. Classical cell culture conditions typically consist of a culturing surface like a cover slip, coated with an adhesive substrate, such as poly-L-lysine (PLL). This, however, discards important structural properties that may have been present in the original microenvironment, which can affect cell growth and further impact the regulation of intracellular mechanisms.

To improve our understanding of how patterned substrates influence adhesion and growth of cells, we have examined neural cell adhesion and differentiation on micropatterned substrates composed of PLL, a common artificial permissive substrate [3-5] as well as growth inhibition on a substrate made from central nervous system (CNS) myelin, known to impair axon regeneration [6]. While we and others have previously used microcontact printing to print PLL, it has not yet to our knowledge been applied to growth inhibitory molecules such as CNS myelin. Myelin, which forms a protective sheath surrounding axons, is composed of many proteins and lipids [7-9]. Some myelin-associated proteins exhibit inhibitory properties that restrict axonal regeneration when nerves are damaged. The study of these molecules in vitro has become a useful tool for investigating axonal regeneration in response to injury as well as numerous neurodegenerative diseases like multiple sclerosis [10-13]. We therefore have developed a protocol for patterning myelin on coverglass using microcontact printing in order to advance our understanding of process outgrowth inhibition in vitro.

We demonstrate, using primary neuronal culture and microcontact printing that neurons adhere to and polarize on diverse patterned environments. While neural lineage cells preferentially adhere to high concentration micropatterned PLL lines, COS7 cells exhibit a concentration-dependent response, favoring low over high concentrations of PLL. Furthermore, we demonstrate that microcontact printing can be used to print coverglass with myelin to study myelin-mediated inhibition of process outgrowth.

## Results

### Control of neuronal morphology by microcontact printed PLL

We first reproduced demonstrations that PDMS stamps can be reliably used to print peptides onto glass surfaces [3-5,14]. For this, we used fluorescein-conjugated-PLL (FITC-PLL) to confirm that microcontact printing is an efficient method for protein transfer to the glass surface (Figure 1). We used different patterns (Figure 1A, D), lines and grids, to examine if cells would adhere to and follow a range of patterned substrates. Primary hippocampal and cortical neurons firmly adhered to patterned PLL (1 mg/mL) and their neurites, visualized using cytoskeletal markers, closely followed the patterns printed in PLL (Figure 1B, C and E, F). An octagonal grid pattern (Figure 1D), with nodes of 20 μm diameter was designed to allow a single neuronal cell body to adhere to each node (Figure 1D). In Figure 1E and F neurons can be seen with their cell bodies positioned within the nodes and the outgrowth of their long processes appears to have been guided by the patterned substrate. Thus, microcontact printing of PLL can be used to control the distribution and morphology of cultured neurons.

**Figure 1:** **Microcontact printing guides neuronal morphogenesis (A) Shown on top is the silicon wafer with dimensions that are compatible with neuronal cell somata i.e., 10 μm wide lines separated by a pitch of 60 μm.** Bottom half of panel shows an example of FITC-conjugated PLL lines printed onto coverglass. In all other cases unconjugated PLL was used. **(B)** Primary hippocampal neurons plated on micropatterned PLL and immunostained for neuron-specific beta-III tubulin. **(C)** Primary cortical neurons plated on micropatterned PLL and stained for F-actin. **(D)** Wafers with octagonal patterns designed to support a single neuronal cell body at each node. **(E, F)** Primary hippocampal neurons plated on micropatterned PLL and immunostained for beta-III tubulin. These neurons position their cell bodies at the nodes and their neurites extend outward, guided by the patterned PLL.

### Micropatterned PLL does not prevent neuronal polarization

We next examined whether this morphological constraint would impair the polarization of neurites into axons and dendrites. For this, we plated neurons onto micropatterned PLL and cultured them for five days. Despite the strict morphological shaping imposed by patterned PLL, Tau-1 and MAP-2 immunostaining to distinguish axons and dendrites respectively revealed no apparent impairment in polarization (Figure 2). Interestingly, the axons can be seen to more closely follow the patterned PLL whereas many MAP-2-positive dendrites are observed to extend outside the defined zones beyond the patterned substrate, suggesting that dendrites may be less strictly guided by adhesive interactions or may be able to secrete extracellular matrix proteins that permit their adhesion to non-printed areas of the glass.

**Figure 2:** **Polarization of neurons growing on micropatterned substrates. (A)** Hippocampal neurons cultured on micropatterned PLL and immunostained for axonal (Tau-1) and dendritic (MAP2) proteins. **(B)** Zoomed image of neuron in **A**. **(C)** Tau-1 immunostaining shows axons closely follow the patterned lines. **(D)** MAP2 immunostaining reveals that dendritic processes can be guided by the substrate, but are also regularly found extending on unpatterned glass. Pattern consists of intersecting 20 μm wide stripes spaced 420 μm apart.

### Microcontact printed PLL regulates the growth of cells with diverse morphologies

We next investigated how patterned PLL might influence the morphologies of cell types with different inherent tendencies to exhibit complex morphological elaboration. For this, we used Oli-neu cells, an immortalized cell line capable of differentiating into immature oligodendrocyte-like cells in vitro [15], and COS7 cells, an immortalized fibroblast line. We used a stamp consisting of parallel lines to print high-concentration (1 mg/mL) FITC-PLL lines on to a background of unconjugated PLL at low-concentration (1 pg/mL) (Figure 3A and 3D) [16]. We found that, similar to neurons, the smaller cell bodies of Oli-neu cells appeared to prefer sites of high concentration PLL and their elaborate processes were aligned with the patterned substrate (Figure 3B, 3C). By contrast, the larger COS7 cells adhered to areas containing lower concentrations of PLL, avoiding the intervening high concentration lines (Figure 3E, 3F). Moreover, the preferential distribution of COS7 cells to the areas with low concentration of PLL is independent of the fluorophore used, as a similar preference was observed when FITC was replaced with DyLight549-conjugated PLL (Figure 4A, B) [17].

**Figure 3:** **Morphological shaping of Oli-neu and COS7 cells by micropatterned PLL (A, D) High concentration (1 mg/mL) FITC-conjugated PLL lines were printed on top of a low-concentration (1 pg/mL) lawn of unconjugated PLL. (B, C)** Oli-neu cells adhered preferentially to the high concentration lines, **(E, F)** COS7 cells showed a preference for the low-concentration PLL regions. **C** is a high magnification image overlaying FITC-PLL (green) from **A** and Oli-neu cells stained with rhodamine-phalloidin (red) for actin from **B**. **F** is a high magnification overlay of FITC-PLL and phalloidin-stained COS7 cells. Scale bars are 60 μm.

**Figure 4:** **Adhesion of COS7 cells on micropatterned PLL.** Schematic representation **(A)** of the three different conditions used: (1) low concentration unconjugated-PLL lawn (1 pg/mL; green) and high concentration DyLight549-conjugated PLL lines (1 mg/mL; red), (2) high concentration DyLight549-conjugated PLL lines (1 mg/mL; red), and (3) low concentration lawn of unconjugated-PLL (1 pg/mL; green). **(B)** Cells seeded onto the first substrate adhere to the low-concentration lawn of PLL avoiding the high-concentration red PLL lines. **(C)** Cells seeded on the second substrate in the absence of a low concentration PLL lawn adhere to high-concentration red PLL lines. **(D)** Cells seeded onto low concentration PLL lawn (1 pg/mL) adhere and display a typical flat morphology. COS7 cells were stained for F-actin. 10 μm wide lines separated by a pitch of 60 μm. **(E)** Quantification of COS7 cell area overlapping printed PLL lines under the conditions schematized in **A**.

In our patterned substrates with 10 μm wide lines printed at 60 μm intervals, 16.7% of the total area of the coverslip is printed with high-concentration PLL. Consistent with their avoidance of high-concentration lines, we found that only 10.2 ± 1.0% of the total area of the COS7 somata and processes grew on the printed lines, significantly less than chance (n = 88 cells in 20 fields; Figure 4E).

The avoidance of the high concentration PLL stripes by COS7 cells reflects either a negative signal from the high concentration stripes or a relative preference for the lower concentration zones. One potential negative aspect of the stripes we used might be that they were simply too narrow to accommodate growth of these large cells. Alternatively it is possible that at these high concentrations PLL may serve as an effective repulsive substrate for COS7 cells. To investigate this, we attempted to grow COS7 cells on high concentration PLL stripes without a carpet of low concentration PLL in the intervening gaps (Figure 4C). Under these conditions, COS7 cells adhered to and extended upon the high concentration PLL stripes (37.8 ± 7.1% overlap, n = 58 cells in 8 fields), showing a strong inclination for growing on these stripes rather than the gaps in between the stripes despite the space constraints of the narrow stripes which covered only 16.7% of the coverslip surface area.

This demonstrates that high concentration PLL, far from inhibiting growth, is actually able to serve as a permissive substrate capable of guiding the adhesion and growth of COS7 cells. The narrow dimensions of the PLL stripes are also not an impediment to healthy growth of the cells. Furthermore, when COS7 cells were plated on a simple lawn of low concentration PLL, adsorbed at 1 pg/mL, they also adhered and grew, indicating that this very low concentration was adequate to support growth on its own and the ability of the COS7 cells to grow on this substrate did not require the presence of the high concentration stripes (Figure 4A and 4D). Therefore, COS7 cells are able to adhere and thrive on either high- (1 mg/mL) or low- (1 pg/mL) concentration PLL substrates but that they distinguish between these concentrations and select the low-concentration PLL microenvironment when given a choice between the two (Figure 4E; p < 0.001, Student’s t-test). This finding underscores the complex influences that the local molecular landscape can exert on growing cells.

### Microcontact-printed myelin inhibits process outgrowth

Recent work has demonstrated that oligodendrocyte differentiation may be tightly regulated by signals produced by other glial cells present in the CNS [10], however this can be a challenge to study under mixed co-culture conditions due to the possibility of reciprocal signaling [18]. We therefore used microcontact printing to quantify the efficacy of myelin in inhibiting process outgrowth in Oli-neu oligodendrocyte progenitor cell lines [10,19]. Oli-neu cells labeled with Cell Tracker Green CMFDA were plated on coverslips micropatterned with PLL, which forced them to extend their processes in a straight line along the printed stripes (Figure 5A, B). Maximum process extension length was then compared between cells in myelin treated and control cultures. Figure 5C shows that myelin significantly impaired Oli-neu cell process outgrowth (myelin-treated: 23.6 ± 2.0 μm, n = 57 vs. control: 35.9 ± 2.2 μm, n = 50, p < 0.001 Student’s t-test).

**Figure 5:** **Microcontact printed substrates demonstrate inhibition of Oli-neu process outgrowth by myelin. (A, B)** CellTracker Green-positive Oli-neu cells plated onto DyLight549-conjugated-PLL lines alone **(A)** or covered with a myelin lawn **(B)**. **(C)** In the presence of the myelin lawn, cells adhere to the PLL lines but exhibit a significant reduction in process outgrowth. **(D)** Microcontact printed myelin lines immunostained for myelin basic protein (MBP; red). **(E)** Control showing the lack of signal when the primary antibody was omitted. **(F, G)** CellTracker Green positive Oli-neu cells plated onto a PLL lawn printed with myelin lines. **(G)** Cells were treated with Y27632, a ROCK inhibitor. **(H)** Cells treated with Y-27632 show enhanced outgrowth compared to the untreated cells.

We next chose to print the protein-enriched fraction of CNS myelin [20] to study myelin inhibition of Oli-neu outgrowth. The crisp pattern of myelin basic protein (MPB) immunoreactivity on stamped coverslips demonstrates that myelin proteins can be efficiently patterned by microcontact printing (Figure 5D, E). Oli-neu cells plated on a carpet of PLL stamped with lines of myelin tend to avoid adhering to or extending upon the myelin stripes, providing further evidence for an inhibitory action of myelin on this oligodendrocyte progenitor cell line (Figure 5F).

Myelin-mediated growth inhibition is believed to involve signaling through the Rho-associated protein kinase (ROCK). Y-27632 is an inhibitor of the ROCK family of protein kinases [21]. Treatment with Y-27632, enhanced oligodendrocyte extension despite the presence of the myelin lines (Figure 5G, H; Y-27632: 68.0 ± 2.0 μm, n = 553 processes vs. no treatment: 42.1 ± 1.2 μm, n = 383 processes, p < 0.001 Student’s t-test). Similar induction of Oli-neu differentiation through the blockade of ROCK has been demonstrated previously [22,23]. Taken together, we demonstrate that microcontact printing can be reliably used to print proteins and protein mixtures onto glass surfaces. We also show that these printed proteins are biologically active and can be used to direct cell morphology and process outgrowth.

## Discussion

Our data demonstrate that microcontact printing is a reliable method for printing growth-permissive and inhibitory proteins on cell culture surfaces. Using PDMS wafers with different geometries, we show that micropatterning of the PLL substrate is an effective way to control the morphologies of neurons in culture. This can be particularly useful in experiments where it is necessary to separate axonal and dendritic compartments of neurons for immunocytochemical or biochemical analyses. We also demonstrated that other cell types such as Oli-neu and COS7 cells exhibit different preferences for PLL substrates. Our discovery that COS7 cells have an unanticipated preference for low concentration over high concentration PLL substrates when provided with the choice in vitro, provides an important insight into how PLL interacts with cells and lays the groundwork for future investigation into the underlying signaling mechanism.

The disparate responses to micropatterned PLL of the various cell types used in the current study provide important insights into the role of the local microenvironment in regulating cell morphogenesis. Similar to neurons, smaller Oli-neu cells adhered and extended their processes along patterned PLL. Larger diameter COS7 cells, however, only chose to grow along high concentration PLL when a low concentration PLL alternative was not provided. This signifies that small differences in local cues are able to tune cell outgrowth in a manner that differs by cell type. Thus such parameters must be considered in designing biomaterials compatible for nerve repair. Similar local control of morphogenesis has been shown to promote precursor cell differentiation in vitro [24]. In that report, the authors showed that populating cell cultures with 10 μm microspheres, a size comparable to the OPC cell body, promoted OPC differentiation into myelin forming cells. We and others have also shown that artificial substrates can be engineered and rationally designed to trigger functional hemisynapse formation by neurons onto biocompatible surfaces [25-27].

In addition, we show for the first time, that a CNS oligodendrocyte cell-derived extract, enriched for myelin proteins can be reliably contact microprinted and used as a functional substrate to study how the microenvironment regulates process outgrowth. This promising approach offers a straightforward in vitro model system in which to examine cellular responses to local growth-inhibitory molecules and to test candidate therapeutic interventions by which to overcome this inhibition. Since myelin growth inhibition is considered a major hurdle to nerve repair following CNS injury, our in vitro model for process outgrowth could be useful in drug screens to identify potential therapeutics that could help mitigate barriers to nervous system regeneration.

## Conclusions

Microcontact printing of growth promoting substrates can be used to examine substrate preferences exhibited by various cultured cells and to guide the morphological elaboration of complex cells like neurons and oligodendrocyte precursors. In addition, micropatterning of growth inhibitory factors such as CNS myelin is useful for examining at a subcellular level how specific cell types respond to such cues and how pharmacological treatments may alter this inhibitory response.

## Methods

All chemicals were purchased from Sigma Aldrich unless specified otherwise.

### Wafer microfabrication and PDMS stamp preparation

Wafers with microsized features were fabricated, as described earlier [3]. Briefly, silicon wafers were cleaned sequentially with acetone, 2-propanol and distilled water, then dried with a gentle flow of nitrogen and left on a hotplate for 1 minute. Photoresist was spin-coated onto the wafers for 30 seconds at 3000 rpm and baked for 1 minute at 110°C. Coated wafers were brought into contact with a chromium mask using a contact mask aligner and exposed under UV light. Polydimethylsiloxane (PDMS) stamps were made by mixing the PDMS elastomer (Dow Corning) from a Sylgard 184 kit with curing agent at a ratio of 10:1 (w/w) and stirred for ten minutes. The solution was poured onto the silicone master with different relief patterns etched into it (wafers) and left standing for 1 hour to remove the bubbles generated during the stirring. The mix was then cured at 60°C for 12 hours in an oven and the molded stamps were then carefully removed from the silicone master.

### Microcontact printing (soft lithography) procedure

PDMS stamps were sterilized under UV lights for 15 minutes. As described earlier [3], prior to PLL loading, the PDMS stamps were immersed in 20% sodium dodecyl sulfate (SDS) for 10 minutes, rinsed with water and air-dried using a high pressure nitrogen stream. Stamps were then incubated for 2 hours with PLL (1 mg/mL), aspirated and then excess solution was removed with a high pressure nitrogen stream. For printing PLL, coverslips were pressed against the inked PDMS stamps and pressure was sustained for a few seconds. In Figure 1A and Figure 3 FITC-conjugated PLL was used to print lines on coverglass. DyLight 549-conjugated PLL was used in Figure 4 and Figure 5A and B. For all other experiments unconjugated PLL was used.

### Microcontact printing of myelin

Myelin extracts were prepared from the bovine brain as previously described (Igarashi et al. 1993). After clarification of the myelin extract by centrifugation at 400,000 g, the detergent was removed by dialysing with phosphate-buffered saline.

To create a PLL lawn on the coverslip, PLL solution was applied for 4–6 hours, and then coverslips were washed with water 3 times. Coverslips were left to dry overnight in a laminar flow hood. Myelin was applied on PDMS stamps and left for 1–2 hours, after which excess was removed using a stream of nitrogen. Immediately afterwards, PLL-coated coverslips were printed using the myelin-coated stamp as above. After applying pressure for 60 sec the coverslip was removed and left to dry at least 3–4 hours or longer.

### Cell culture

Low-density hippocampal cultures were prepared from embryonic day 18 (E18) Sprague Dawley rats as described earlier [28]. In brief, pregnant rats were sacrificed by CO2 intoxication. The fetuses were removed, decapitated, and the heads were transferred into culture dishes containing Hank’s Balanced Salt Solution (HBSS, Invitrogen). The hippocampi were dissected, transferred to 15 mL conical centrifuge tube, trypsinized for 15 minutes at 37°C, washed three times with pre-warmed HBSS and cells were finally resuspended in Neurobasal medium (containing Gibco supplements; B27, L-glutamine, and penicillin/streptomycin) after a brief centrifugation at 1000 rpm. The cells were then plated at moderate density (40,000 cells/well in a 12 well plate), cultured for five days in a 37°C incubator containing 5% CO2, and analyzed for morphology and polarization.

Rat cortical neurons were prepared from embryonic day 17–18 rat cortices [11]. The cortex was dissected, dissociated with trypsin and mechanical trituration, and cultured for 7 days on dishes coated with 0.01% poly-l-lysine (Sigma). Neurons were grown in Neurobasal medium, 2% B27 supplement, penicillin/streptomycin, and 1% glutamine.

Oli-neu cells and COS7 cells were cultured as described previously [29,30]. Oli-neu cells were treated overnight with 2 μM Cell Tracker Green CMFDA (5-chloromethylfluorescein diacetate) (Molecular Probes, C2925) then reseeded at 80,000 cells/well onto stamped coverglasses in a 12-well plate. Oli-neu cells were serum-starved with 0.1% horse serum in DMEM to initiate differentiation, and treated with either vehicle control or 10 μM Y-27632 (EMD Millipore, 688001) for 24 h. Cells were then fixed with 2% PFA and mounted on slides.

All procedures involving animals were approved by the Animal Care Committees of the Montreal Neurological Institute and McGill University.

### Immunocytochemistry

For hippocampal and cortical neuron immunostaining, cultured cells were briefly rinsed in pre-warmed phosphate buffered saline (PBS, Invitrogen), fixed for 10 minutes in 4% paraformaldehyde (PFA) in PBS, washed 3 times for 10 minutes in PBS, permeabilized for 5 minutes in 0.1% Triton X-100 and blocked in 5% bovine serum albumin (BSA) for 60 minutes. The following primary antibodies diluted in 5% BSA/PBS for 1 h at room temperature were applied at the given dilutions: mouse anti-beta-III-tubulin (1:1000, Abcam), mouse anti-tau-1 (1:150, Chemicon), chicken anti-MAP2 (Gene Tex, 1:1000). After 3 washes of 5 minutes each with PBS, species matched fluorochrome conjugated secondary antibodies were applied for 45 minutes. Fluorochrome-conjugated antibodies were applied at the following dilutions Alexa488 (1:400) and Cy3 (1:2000). Excess and unbound secondary antibodies were removed by three washes of PBS (5 minutes each) and the coverglasses were mounted in Aqua-Poly/Mount (Polysciences, Warrington, PA) on glass slides for confocal analysis. Oli-neu and COS7 cell were processed as described earlier [29,30]. To visualize F-actin, rhodamine- or FITC-conjugated phalloidin staining was used.

### Image capturing and analysis

Fixed and immunostained cells were imaged using an Olympus Fluoview FV1000 laser scanning confocal microscope with a 60x PlanApo oil-immersion objective (1.4 numerical aperture) on an IX81 inverted microscope. For double immunostaining, images were acquired via sequential scanning of each individual channel. The acquired images were processed with Adobe Photoshop CS2 and process outgrowth was analysed with NeuronJ, a plugin of the NIH freeware ImageJ software. Two-tailed unpaired t-tests were used for statistical analysis. The graphs show mean ± standard error of the mean. For all conditions at least 40 cells were randomly selected from 3 coverslips each.

## Competing interests

The authors declare that they have no competing interests.

## Authors’ contributions

WB, DRC, and ASD conceptually designed the study. WB performed all experiments. PT provided wafers. PTY made the DyLight 549-conjugated PLL and contributed to the optimization of the micropatterning technique. CAJ performed the myelin experiment. WB, ESR, DRC, and ASD wrote the manuscript with input from all authors. All authors read and approved the final manuscript.
